RETRACTED

# Research on Data Security and Privacy Protection of Wearable Equipment in Healthcare

**DOI:** 10.1155/2021/6656204

**Published:** 2021-02-05

**Authors:** Dawei Jiang, Guoquan Shi

**Affiliations:** ^1^School of Mechatronical Engineering, Changchun University of Science and Technology, Changchun 130000, Jilin, China; ^2^School of Mechatronical Engineering, Changchun University of Technology, Changchun 130000, Jilin, China

## Abstract

With the close integration of science and technology and health, the broad application prospects of healthy interconnection bring revolutionary changes to health services. Health and medical wearable devices can collect real-time data related to user health, such as user behavior, mood, and sleep, which have great commercial and social value. Healthcare wearable devices, as important network nodes for health interconnection, connect patients and hospitals with the Internet of Things and sensing technology to form a huge medical network. As wearable devices can also collect user data regardless of time and place, uploading data to the cloud can easily make the wearable device's system vulnerable to attacks and data leakage. Defects in technology can sometimes cause problems such as lack of control over data flow links in wearable devices, and data and privacy leaks are more likely to occur. In this regard, how to ensure the data security and user privacy while using healthcare wearable devices to collect data is a problem worth studying. This article investigates data from healthcare wearable devices, from technical, management, and legal aspects, and studies data security and privacy protection issues for healthcare wearable devices to protect data security and user privacy and promote the sustainable development of the healthcare wearable device industry and the scientific use of data collection.

## 1. Introduction

Health occupies a pivotal position in people's daily lives. As the saying goes, “The body is the capital of the revolution,” and it is also a health issue. In recent years, with the rapid development of China's economy, living standards have changed dramatically, and health problems are increasingly appealing to the public as a result of population aging. In particular, people living in cities have long-term dietary and irregular diets, subhealth and chronic diseases are gradually becoming younger, and the health of the people is worrying [1–3]. In this context, with the development of mobile medical services, smart wearable medical products have emerged, which combines information technology such as network big data, cloud medical, cloud computing, and medical care institutions to provide users with personalized health. Health and medical information, to remind users to pay attention to their own health, prevents problems before they occur [4]. Although the smart wearable medical product market has been developed very early at home and abroad, it is still in its infancy, in this respect, because the technical problems of the equipment have yet to be developed and, on the other hand, because most users who purchase equipment use equipment. The stickiness is not enough, and there is no explosive growth in the market for the time being.

RETRACTED

Based on this, with the development of smart phones, smart wearable devices such as smart bracelets and smart glasses have gradually entered people's lives and become the new favorite in the market [5]. Among them, mobile medical equipment is the most influential, and smart wearable medical products are a market segment of the wearable market. They are primarily used in the field of healthcare and are used in healthcare, diagnosis and treatment, chronic disease management, and out-of-hospital rehabilitation. The year of prosperity and development will not only monitor the health of users in a timely manner, but also alleviate the shortage of medical resources in China to a certain extent, making the development of the medical field a big step forward [6–8]. As an electronic product, the smart wearable device can be installed in the clothes to be worn or worn on the outside of the human body. It has network connection, sensors, and even touch screen operation technology, and its function design is relatively user-friendly. In the process of use, the smart wearable medical device can record the wearer's pulse, ECG, heart rate, blood lipids, blood pressure, and other health data as well as the state of motion and sleep quality in daily life, and the data of mobile phones, tablets, and other electronic equipment is synchronized, and the health information returned by the healthcare institution is received in time to detect the disease early, prevent and supervise the disease, and achieve the purpose of monitoring the health of the user, preventing the problem [9–12]. In addition, smart wearable devices have a variety of additional features that make it easier for people to produce and live. For example, in addition to monitoring health data such as user movement, sleep, heart rate, and blood pressure, some smart bracelets also have functions such as receiving information, mail, and network payment, which avoids the user's need to frequently check the mobile phone. There are also some smart wearable devices with remote control of cars, household appliances, small projectors, and other functions, which not only bring great convenience to people's lives, but also attract the attention of many college scholars and researchers [13]. At present, many well-known IT brands at home and abroad have invested in the research and development of smart wearable medical products. The main types of products include smart wristbands, smart watches, wrist pulse oximeters, muscle sensors, etc. [14]. Applied research on wearable technology has achieved some results in the medical field. In the treatment of Parkinson's disease, Kita et al. developed a wearable device “Gait-Assist” that can help patients overcome the frozen gait [15]. In terms of detection, Na et al. developed a hearing aid dynamic electromechanical device [16]; in terms of surgical navigation, Rosenthal and Harmsen designed a visual navigation software for cancer tumor resection [17–19]. It can be seen that wearable device applications have many advantages in the medical and health industry, and researchers are turning theory into a real product, and the medical health industry can be expected to be an important market for wearable devices in the future [20, 21]. According to ABI Research, a US research and analysis company, the revenue of wearable wireless medical health equipment is expected to exceed $8 billion in 2019.

RETRACTED

However, in recent years, there have been scandals of data leakage, such as the fact that Fitbit is vulnerable to being acquired by others in the state of network connection, and the network address is easily recognized. Xiaomi, Huawei, Jawbone, and other manufacturers have also experienced data leakage. Some of these wearable devices have been forced to withdraw from the market because of infringement of personal privacy that hinders the development of their products. In addition to technical reasons such as equipment and network, data transmission, privacy awareness is also an important factor affecting data security and privacy protection of healthcare wearable devices [22–24]. Wearable devices can also collect user data regardless of time, place, and occasion and upload data to the cloud, which makes the wearable devices vulnerable to attacks and data leakage. In this way, this paper uses a questionnaire survey to investigate the data security and privacy protection awareness of wearable devices in healthcare, from the awareness of data security capability of devices, data rights subject, and number. According to the awareness of sharing willingness, respect for other people's privacy, data protection, and rights protection, the survey results were analyzed, the main problems were elaborated, and countermeasures were put forward.

## 2. Methods

### 2.1. Wearable Device Classification

Wearable devices are products that use information and communication technology, electronic chip technology, and sensor technology to integrate intelligent design of clothing and equipment that can be worn directly on the body. The device typically uses biosensors to detect the user's physiological indicators in real time and record lifestyles and behaviors such as diet and exercise. To allow detailed investigation of the data collected by the device, the device uses wireless communication technology to upload the data to the Hth server or cloud via a mobile phone or computer for professional analysis. We process data professionally through the program. At present, wearable devices have covered sports detection, personal health management, positioning and navigation, leisure and entertainment, mobile payment, social interaction, and many other fields, which greatly enriched the wearer's perceived experience. Currently, health management and medical-assisted wearable devices are the most popular on the market, with the largest number of products launched, and various types of bracelets, watches, and wristband products occupy more than 80% of the market, and consumers are most concerned about such products. Health management manufacturers use the original professional sports production experience, combined with sensor technology, to provide detection and analysis of environmental indicators (such as air pressure, altitude, and diving depth) such as the state of the sport (such as rate, frequency, and calorie consumption). Manufacturers of medical aids mainly develop portable devices, commercialize medical research results, and provide sophisticated analysis of medical signs such as blood glucose, mandatory rate, and blood pressure. The health and medical sectors are seen as the most promising market for wearable devices. The first reason is that people are paying more attention to health. These products can easily monitor daily exercise and sleep quality. Secondly, they are easy to operate. Learning to use, and with the emergence of new sensors, will introduce more scientific and more humane products in the health and smart market, such as non-invasive blood glucose monitoring equipment. According to the complexity of the technology used by wearable devices, wearable devices can be divided into two categories:

1. The first is a wearable device mainly using a sensor, including a smart wristband, a smart watch, and the like. Such devices can be subdivided into two subcategories based on application functionality: health indicators and motion tracking classes and smartphone-assisted classes. Health indicators and sports tracking products include the Fuelband smart wristband, the Jaebone UP smart bracelet, the Plump bracelet, and the Fitbit Flex smart bracelet. These products mainly use the sensing device to record the user's movement and physical health, and then connect with the intelligent terminal device so that the user can analyze and deeply manage the data to clearly understand their own situation. Smartphone-assisted products include Pebble watches, Galaxy Gear smart watches, and more. These devices are usually used in conjunction with a smartphone to make the game work. The wearer uses the device to perform functions such as making calls, sending and receiving emails, and processing text messages on the smartphone, simplifying the use of the mobile phone.
2. The other is a wearable device that combines human-computer interaction technology, mainly a smart eyewear product. This type of equipment not only uses sensors to collect data, but also uses complex human-computer interaction techniques to enhance the application. Such wearable devices can be attributed to integrated smart terminal types according to application functions, such as Google Glass smart glasses, ReconJet smart glasses, and the like. These devices are usually enhanced after being connected to mobile phones, and use a variety of new human-computer interaction technologies such as new display technologies, voice interaction technologies, augmented reality technologies, and image recognition technologies to meet the user's virtual and realistic experience.

RETRACTED

### 2.2. Significance of Wearable Equipment for Healthcare

#### 2.2.1. Theoretical Significance

Modern information technology has been applied to various development fields, and the healthcare industry that keeps pace with the times is no exception. In recent years, more and more attention has been paid to the construction of information technology. Electronic medical treatment has become popular and has been in the normal operation of medical institutions. The role of substitution provides a lot of convenience for both the hospital and the patient. In recent years, the combination of mobile smart devices and electronic medical care has made mobile medical treatment possible. Today, with the rapid development of “Internet +,” mobile medical has great potential for development, and the number of smart wearable medical products is increasing day by day. We believe that our medical environment will be greatly improved in the future, and the health quality of the people will also have a big boost. Therefore, in order to make the market have a more benign development, it is of great theoretical significance to analyze the willingness to consume smart wearable medical products:

1. At present, most research studies on smart wearable medical products focus on product development, design, and development status. Most of the research methods used are based on questionnaire data and previous literature, and there is not enough persuasive power to explain the research model. Setting, and research on the willingness to consume smart wearable medical products, is rare. Therefore, this paper takes the people who pay attention to their own health status as the research object, and explores the factors affecting the willingness to consume smart wearable medical equipment, so as to explore the deeper connotation of the market and enhance the consumer behavior analysis of smart wearable consumer goods.
2. Wireless network technology is advancing by leaps and bounds and plays an important role in people's daily lives. It can be said that, without the network, we cannot work and live at all. Based on this, the smart wearable medical products provide users with a variety of health information, so users no longer need to go to the hospital to find experts because of some problems in the body, which saves their own time and medical expenses. It has also greatly eased the situation of hospital congestion and shortage of medical resources, and improved the efficiency of medical treatment. Therefore, studying the influencing factors of the willingness to consume smart wearable medical products is helpful to clarify which factors will lead users to adopt certain technologies and enhance the analysis of target customer services.

RETRACTED

#### 2.2.2. The Actual Meaning

The rapid rise of smart wearable medical equipment has had a certain impact on the traditional medical industry. The National Center for Health Information Statistics estimates that more than half of the national medical expenses will be spent on the elderly in 2050, and as the population ages and the chronic disease population increases, medical expenses will also increase exponentially, creating a growing risk of total medical expenses in an aging society. Therefore, researching healthcare can only wear product privacy protection is also responsible for the medical healthcare of the elderly in China, and has certain practical value. (1) Although smart wearable devices have been developed very early at home and abroad, the development momentum has always been insufficient, the market is still in its infancy, and the purchases of products by users are generally low. In recent years, combined with the development of biomedical sensing, Internet of Things, big data, “Internet +”, and other technologies, the market has become active and has good development prospects. Therefore, by studying the factors that influence the consumer motivation of smart wearable medical devices and gaining a deeper understanding of users' product demands, we can make breakthroughs, keep pace with the times, and achieve greater progress. (2) Research on healthcare can only wear the influencing factors of product privacy protection. On the one hand, the research results can be used by investors and manufacturers for reference, so that product technology can be improved to meet the needs of consumers, and it is also beneficial. The producers are further profitable; on the other hand, the research on the influencing factors has certain reference value for the people who pay attention to their own health status, and they can deeply understand the psychological thoughts of the public when purchasing smart wearable devices, thus making self-judgment and rational consumption, improving the correctness and timeliness of independent consumption. Furthermore, research on the market for smart wearable medical products can promote the development of the smart wearable device industry and will also drive the entire medical and health field in China.

RETRACTED

### 2.3. Health and Medical Wearable Devices Data Security and Privacy Protection Problems

Based on the characteristics of data collection and flow of healthcare wearable devices, combined with China's national conditions, the problems in data security and privacy protection of healthcare wearable devices will be summarized from three aspects: technical security, data management, and laws and regulations.

#### 2.3.1. Technical Safety Issues

Healthcare wearable devices are highly dependent on IOS and Android systems, and system vulnerabilities are easily attacked by hackers, causing private data to leak. In the process of data collection, due to the lack of control over devices and data permissions, users cannot choose to shut down a sensor individually or cancel data collection, making it difficult to authorize the viewing and use of data. In the process of data transmission, the healthcare wearable device's MAC address is basically fixed and uses a relatively simple data format (such as JSON) to directly transfer the collected data values or pictures, and lacks multiple encrypted data blurring measures. Others are easy to connect with devices and get data information.

#### 2.3.2. Data Management Issues

Healthcare wearable devices are developing rapidly. The data transmission formats, encryption and confidentiality, integrated platform interfaces, and data transmission protocols generated by various devices lack uniform industry standards, and a series of problems such as information silos and privacy protection have emerged. This is not only easy to cause leakage of user health information, causing health discrimination, but also endangering national security and stability.

RETRACTED

#### 2.3.3. Legal and Regulatory Issues

The wearable device industry is a newly emerging and fast-growing industry. The country currently lacks policies and regulations on data security and privacy protection for wearable devices, especially healthcare wearable devices, once wearable device manufacturers sell user data privately. It will be difficult to pursue their responsibilities according to law. In addition, there is no uniform industry standard for the data format and content collected by healthcare wearable devices, which brings great difficulties to the storage and management of data, which is not conducive to the integration and utilization of data.

## 3. Experiments

### 3.1. Research Methods

#### 3.1.1. Literature Research Method

This was through research on domestic CNKI, Wanfang, Weipu, foreign PubMed, and other literature databases to access health medical wearable devices and their research literature related to data security and data privacy, to analyze the current relevant research progress, healthcare wearable devices. The proposed data security and privacy protection methods summarize the solutions and countermeasures for data security and privacy leakage in the development and application of healthcare wearable device data.

#### 3.1.2. Questionnaire Method

Questionnaires were used to conduct research on experts and scholars in the field of medical informatization and the general public. The data security and privacy protection awareness of healthcare wearable devices was taken as the main content of the survey, revealing the user's data security for healthcare wearable devices. Privacy awareness and ethical respect were taken as the main content of the survey.

### 3.2. Research Data

From May 2017 to May 2018, questionnaires were conducted on the awareness of data security and privacy protection of wearable medical devices for teachers and students of local medical colleges. According to the different titles of the respondents, 235 questionnaires were distributed by stratified sampling method, and 223 questionnaires were recovered, with a recovery rate of 94.9%.

Through the research and analysis of the influencing factors of consumers' willingness to wear products privacy protection in healthcare based on personal concern, and after classifying and integrating the variables, the variables are summarized as the following three factors: personal characteristics, personal health status, and personal attitudes towards healthcare only wearing products privacy protection. In three aspects, the specific influencing factors can be defined, as shown in Table 1.

RETRACTED

We will make personal characteristics and personal health factors to make the individual's attitudes to the healthcare only wear product privacy protection factors, personal attention to health data, and personal attention to healthcare concerns. Factor analysis yields a significant degree of influence on the willingness to protect privacy.

## 4. Discussion

### 4.1. Health and Medical Wearable Device Data Survey

67.8% of the respondents believed that the data should belong to the users themselves, far higher than the medical service institutions responsible for docking and the relevant government departments. In addition, 34.1% of the respondents thought that the subject of right should be the user himself. 26.5% and 13.1% thought that the subject of right could be the specialist of diagnosis and treatment and the manager of the medical service organization responsible for docking, respectively. 9.3% of the respondents thought that the subject of right should be the user himself. 26.5% and 13.1% of the respondents thought that the subject of right could be the specialist of diagnosis and treatment and the manager of the medical service organization responsible for docking. From this, we can see that most of the respondents believe that the data owners of wearable medical equipment are users themselves, and they have the right to view and modify the data. Few respondents believe that the data owner is the relevant government sector of the country. If the relevant government department wants to view and change your data, they should obtain user permission beforehand. There are great differences in the cognition of the subjects responsible for data disclosure. The specific results are shown in Figure 1.

Due to the lack of mandatory protection measures and uniform standards, data is easily intercepted and tampered with. Therefore, healthcare wearable devices should apply multiple data encryption technologies at the device terminals and the cloud. Setting the data content protection level increases the flexibility of operating permissions and controls data protection costs. This paper divides the data privacy protection of healthcare wearable devices into five categories (Table 2). Combined with the impact of data privacy disclosure on the country and individuals and the value of data, the privacy protection level is divided into three levels: A, B, and C. The privacy protection is further divided into 2 levels (A+ and A; B+ and B).

There are specific requirements at each level. The A-level requirement is to adopt the most stringent encryption and authentication protection technology. Non-legal permission prohibits collection, viewing, and use, and A+ and A-level legal supervision and punishment are different. The privacy protection level is A+ Class I data and privacy protection. Class II data of level A needs to be de-sensitized; the requirement of level B is that, after the user's informed consent, the authorized object views, uses, and modifies the data within the specified service and scope, and the identity authentication technology should be used to guarantee the authorized identity. The rationality, in which the B+ level data should meet the clinical data protection standards, the B-level privacy data can be opened in combination with the clinical situation; the C-level requirement is that the user can independently share the V-type data in the healthcare wearable device terminal, but provide ethics A risk statement that respects the privacy of others.

RETRACTED

For the data sharing willingness of healthcare wearable devices, whether they want to synchronize their collected data to the cloud, whether they want to upload their own data in real time, and whether their own behavior data and environmental data are reasonable, the survey results are shown in Figure 2.

47.1% of the majority of respondents are more willing to share their own data, and it is considered reasonable to share personal behavior data and environmental data, but data sharing should be carried out with their own informed consent or authorization. Users who use healthcare wearables not only lack privacy awareness, but also easily ignore respect for the privacy of others. When the device collects data, it not only collects personal vital signs data, but also collects data of the surrounding environment. The device has recording and photo/video recording capabilities, and in the process it also captures the privacy data of the people around you.

### 4.2. Data Security and Privacy Protection Measures for Healthcare Wearable Devices

#### 4.2.1. Technical Level

Because the data of wearable equipment in healthcare covers a wide range of fields, the link of data flow is complex, the mobility of equipment, and the small size of equipment, it is necessary to carry out technical protection measures of wearable equipment in healthcare based on the premise of law and management. You need to establish a hierarchically categorized data management and control model that includes multi-level assurance of data content protection levels and data flow links. To control data access, you need to actively use multiple data encryption and identity authentication technologies. In addition, the recognition ability of scene switching and the remote control ability of remotely clearing and missing reminders of data should be optimized.

RETRACTED

#### 4.2.2. Management Level

To improve the management of data security and privacy protection of wearable equipment in healthcare, we should first prevent abuse of power by relevant government departments, secondly, we should step up the introduction of national data protection standards and strengthen the construction of industry self-discipline, thirdly, we should improve the responsibility traceability mechanism in the process of data use to ensure the reasonable access of data, and finally, we should increase the training of healthcare big data hiding. For private protection professionals to promote healthcare wearable equipment, data security and privacy protection research and work are also important.

#### 4.2.3. Legal Level

At the legal level of data security and privacy protection of wearable healthcare equipment, China should establish a specific legal system for personal data protection, clarify the scope of data protection of wearable healthcare equipment, and then make legal provisions for data security of wearable healthcare equipment stored in big data cloud platform to achieve mandatory wearable healthcare data. Legal construction of security and privacy protection are also established.

## 5. Conclusions

The core issue of data security and privacy protection is data. Although there are a certain number of related researches on data security and privacy issues of wearable devices, most of them are for general wearable devices. Healthcare wearable devices are rarely used as the key analysis objects, and the collected data are not completely flowed. The process is the main content of privacy research. In addition, the research on data security and privacy protection of wearable devices mostly focuses on a certain level, especially the algorithm and network security at the technical level. There are a few discussions on privacy issues such as management, lack of integrity, and comprehensiveness. Research on data security and privacy protection for healthcare wearable devices has established a systematic, multidimensional system framework and designed different levels of specific protection against data characteristics and mobile links, and different types. You need to establish privacy standards for your data. In combination with the responsibility of the participating national governments, industry producers, hospitals, third-party participating institutions, and individuals, the roles and responsibilities of different role entities should be used to protect the data security and privacy of healthcare wearable devices. Healthcare wearable devices are developing rapidly, and the data security and privacy issues involved in their domain specificities are more complex and directly related to personal life safety and even national security. Therefore, it is more urgent to solve this problem, and it is necessary for many parties to participate in efforts to establish a reasonable and effective privacy protection mechanism.

RETRACTED

## Figures and Tables

**Figure 1:** Analysis of data ownership cognition of healthcare wearable devices.

**Figure 2:** The survey object's rationality on shared behavior and environmental data.

**Table 1:** Specific analysis of influencing factors.

Dependent variable	Independent variable		
	Variable attribute	Serial number	Variable name
Would you like to know about healthcare wear privacy issues?	Personal characteristics	A1	Gender
		A2	Age
		A3	Education level
	Personal health	B1	Abnormal health indicators
		B2	Subhealth
	Personal wear attitude	C1	Attention to wear
		C2	Thinks smart wear is the trend
		C3	Treatment of subhealth issues
		C4	Discover and treat health as early as possible

**Table 2:** Healthcare wearable device data privacy protection level division table.

Category	Criteria for the classification	Data content	Privacy level
1	Data that pose a threat to national public safety	Integrate associated healthcare wearable device data	A+
2	Data that directly identify the user's identity	PII (including all healthcare wearable device data) PHR	A
3	Data that are closely related to the health of the user	Data on vital signs, health warnings, and medical records	B+
4	Data that are highly relevant to user health and identity	Sports behavior, emotions, etc. data	B
5	Data that indirectly affect a user's health	Sports behavior, emotions, etc. data	C

## Data Availability

No data were used to support this study.
